The article "A Mutagenesis Assay for Reporter Gene Screening Using Partially Degenerate Oligonucleotides of the Tandems NNT and NNC" was published in 2015. Journal: Biomed Res Int.

# A Mutagenesis Assay for Reporter Gene Screening Using Partially Degenerate Oligonucleotides of the Tandems NNT and NNC

**DOI:** 10.1155/2015/950873

**Published:** 2015-06-18

**Authors:** Huifen Xu, Cuilan Zhou, Andy K. Zhang, Wen Li, Jia Zhang, Kai Li

**Affiliations:** ^1^Department of Molecular Diagnostics and Biopharmaceutics, College of Pharmaceutical Science, Soochow University, Suzhou 215123, China; ^2^Department of Human Anatomy, University of South China, Hengyang 421001, China

## Abstract

Not all proteins are tolerable to mutations. Whether a specific protein can be a mutable target is of importance in the biotechnology and pharmaceutical industry. This study reported a novel mutagenesis assay using tandem NNT and NNC oligonucleotides to test the mutability of a candidate gene. These two tandem oligonucleotides avoid the risk of forming nonsense mutations and render flexibility of truncating or expanding the insertion size. As a reporter gene, ZeoR (zeocin resistance gene) was confirmed to have a high tolerance for mutagenesis by this new assay.

## 1. Introduction

The development of TALENs and CRISPR/Cas9 systems, together with the well-recognized ZFNs, renders gene editing technology a hot topic in genome modification used in both fundamental research and human gene therapy [1–8]. Currently, the majority of the related studies employ gene editing technology aimed at modifying genes or genomes in cells or in model organisms. The most attractive application of gene editing technology in human gene therapy is largely restrained by the lack of sensitive methods to evaluate the off-target effects of genetically engineered nucleases.

From the therapeutic point of view, the off-target effects of genetically engineered nucleases are tantamount to the side and toxic effects of small molecule drugs. As genetically engineered nucleases are the most promising large molecule candidates in human gene therapy, minimizing the off-target effects is the prerequisite for their application in human gene therapy. Some assays, such as single-strand annealing assay, can be used to evaluate the enzymatic activity of genetically engineered nucleases but are too insensitive to analyze their off-target effects [9]. Recently, we tested whether *β*-galactosidase and KanR could be used in the development of assays for off-target effects. We recognized that the *β*-galactosidase-based assay had unacceptably high false positives and negatives, and the KanR-based assay showed a sequence-specific intolerance to mutagenesis [10]. It seemed that an ideal reporter gene for assays in evaluating off-target effects should fulfill two requirements: high tolerance to mutagenesis and little to no leakage in respect to false positives.

Established methods in mutability analyses and mutagenesis assays have been successfully employed in the evaluation of how mutable a gene or genome is regarding the phenotype-genotype relationships and how potential mutagens cause gene mutations [11–13]. For screening or testing the mutagenesis effect of potential mutagens, a number of in vitro and in vivo assays have been developed and widely used, such as deep sequencing and mismatch Cel 1 or T7 [14–21]. In general, these aforementioned methods are useful in evaluation of mutation spectra of either a gene, a genome, or a mutagen. But these methods are not designed for the analysis of the tolerance of a gene.

ZeoR was chosen in this study since it can be used as a select gene for both prokaryotic and eukaryotic cells [22–24]. Two types of tandem oligonucleotides, NNC and NNT, were used as inserts in the mutagenesis test. Highly heterogeneous products from these mutagenesis analyses were identified. The mutants consisted of various lengths of inserts with no bias in their base uses at each degenerate site. Furthermore, the dual drug resistance of the plasmid pZAmpB simplified the screening of any potential false positives. The usefulness of the mutagenesis tolerance assay in screening reporter genes was confirmed with the usage of these tandem nucleotides in mutants and further mutants with a series of specific sequences.

## 2. Materials and Methods

The plasmid of pPICZ was purchased from Thermo Fisher Scientific, Inc. (Waltham, USA). Plasmid PMD-19 was purchased from TaKaRa (Dalian, China). Oligonucleotides used in the study were synthesized by GENEWIZ, Inc. (Suzhou, China). All restriction endonucleases except BaeI were the products of New England Biolabs, Inc. (Massachusetts, USA) and other enzymes including Pfu and Taq polymerases and T4 DNA ligase were the products of Thermo Fisher Scientific, Inc. (Waltham, USA).

## 3. Methods

### 3.1. Development of a Dual-Resistance Plasmid for Mutagenesis Assay

Overlap extension PCR was used in the construction of plasmid pZAmpA and pZAmpB (Figure 1(a)). The plasmid of pZAmpA was created from PMD-19 by the replacement of the lacZ cDNA by the zeocin-resistance gene from pPICZ. The pZAmpA plasmid was designed to contain both zeocin- and ampicillin-resistance genes. The BaeI recognition site behind the start codon ATG of zeocin-resistance gene was to be further introduced into pZAmpA which would subsequently be subjected to mutagenesis. Two restriction sites of HindIII and EcoRI resided within the BaeI site (Figure 1(b)) for the mutants' initial screening with colony PCR.

PCR extension conditions have been described elsewhere in detail [25]. In short, primer extension was carried out for 30 cycles with 30 s denaturation at 95°C, 30 s annealing at 58°C, and 30 s extension at 72°C. The primer extension reaction was performed in a total volume of 25 *μ*L with PMD-19 or pPICZ as the template reaction system, 0.2 mM deoxynucleotide 5′-triphosphate (dNTP), 10 mM of both sense and antisense primers, 2.5 *μ*L of the 10x Pfu buffer with MgSO_4_, and 0.625 U Pfu polymerases.

### 3.2. Insertion Mutagenesis with Degenerate NNT and NNC Oligonucleotides

The golden gate cloning strategy was used to test the mutability of the zeocin gene in the plasmid of pZAmpB. Golden gate cloning takes the advantage of Type IIs restriction enzymes of cutting DNA outside of their recognition sites. Combining Type IIs restriction enzyme and DNA ligase, golden gate cloning allows the cloning of nonpalindromic overhangs [26]. The vector pZAmpB was first digested with BaeI and then gel purified. Two types of degenerate oligonucleotide inserts, the tandem NNT and the tandem NNC, were tested. This subcloning strategy is illustrated in the Figure 1. The sequences of the tandem inserts are shown as follows:

 NNT+: 5′-NNTNNTNNTNNTNNTNNTNNTNNT
 GCCAA-3′,
 NNT−: 5′-ANNANNANNANNANNANNANNAN
 NCATAG-3′,
 NNC+: 5′-NNCNNCNNCNNCNNCNNCNNCNN
 CGCCAA-3′,
 NNC−: 5′-GNNGNNGNNGNNGNNGNNGNNGN
 NCATAG-3′.

Oligonucleotide inserts were annealed to form dsDNA before ligation reaction. A pair of NNT+ and NNT− oligonucleotides was added to the 10 × L annealing mix at 100 pmol each. The annealing mix was heated at 95°C for 5 min, then cooled down to the temperature of 37°C at the speed of 0.5°C/min, and then stored the annealing product at 4°C. The pair of NNC+ and NNC− oligonucleotides was treated similarly.

The ligation reaction was performed in a total volume of 10 *μ*L using the annealed oligonucleotide pairs and gel purified vector fragment. Each ligation reaction mix contained 20 ng of vector, 1 *μ*L T4 DNA ligase, 40 ng of each dsDNA, and 1 *μ*L 10 × T4 DNA ligase buffer. After ligation at 22°C for 40 minutes, all of the reaction solution was applied in transformation using DH5*α E. coli* strain. Colonies were picked from overnight growth on the zeocin plate for further PCR confirmation analysis and commercial DNA sequencing analysis.

### 3.3. Mutagenesis Using Nondegenerate Oligonucleotides

Two types of nondegenerate oligonucleotides were tested: those with a size divisible by 3 and those with a size not divisible by 3 (Table 4). These nondegenerate oligonucleotides included some of the targets of TALENs and CRISPR/cas9 that were designed for future studies. These nondegenerate oligonucleotides were subcloned using double overhangs and ligated with the vector in the presence of T4 ligase to simplify the procedure.

### 3.4. Statistical Analyses

Fisher's exact test was performed using SPSS19.0 (SPSS, Chicago, IL, USA).

## 4. Results

### 4.1. Development of a Dual-Resistance Plasmid for Mutagenesis Assay

A plasmid containing both ampicillin- and zeocin-resistant genes was subcloned. This new plasmid was first confirmed in LB plates with ampicillin and zeocin, respectively, and then by sequencing analysis (Figure 2).

The plasmid was further modified by integrating a BaeI site between the first and the second triplets of the ZeoR coding sequence. As shown in the Figure 2, two 6-base restriction sites were resided within the BaeI site: the HindIII and EcoRI.

### 4.2. Insertion Mutagenesis with Degenerate NNT and NNC Oligonucleotides

Both tandems (NNT)_8_ and (NNC)_8_ have successfully yielded mutated constructs with zeocin-resistance retained. Both of these degenerate oligonucleotides were able to form a large number of colonies.

Heterogeneous mutated constructs were identified from the tandem NNT and NNC degenerate oligonucleotides (Figure 3). For the twenty colonies sequenced for these two oligonucleotides, 14 out of 20 and 17 out of 20 colonies contained either a truncated or expanded tandem of NNT and NNC oligonucleotides, respectively. The remaining colonies were unsuccessful in sequence analysis.

Regardless of the size of the inserted tandem oligonucleotides, the degenerate bases were randomly employed by the mutated constructs (Table 1). At each of the degenerate sites, all four types of nucleotides (A, T, C, and G) were used in the successfully sequenced 31 colonies. Fisher's exact test showed that there was no bias in the nucleotide use at any of the degenerate sites (*P* > 0.05 for both tandem NNC and NNT oligonucleotides).

For the two tandem oligonucleotides, the inserted fragment showed different heterogeneities. The NNT sequences were less random in comparison to those of NNC (Table 2). Interestingly, these different heterogeneities showed statistical significance. Although all possible appearing amino acids were identified in the collection of either the 14 or the 17 positive colonies, Fisher's exact was unable to analyze their randomness due to their limited number.

### 4.3. Mutagenesis Using Nondegenerate Oligonucleotides

A total of 5 nondegenerate oligonucleotide pairs were tested by inserting them into the site right after the initiate codon of ZeoR gene. As shown in Table 4, mutants in the size not integer divisible by 3 inserts only grew in ampicillin plate, and all mutants in the size integer divisible by 3 inserts grow in both ampicillin containing plates and in zeocin containing plates. These mutants are highly heterogeneous in their insert lengths and sequences, indicating that the mutability of zeocin enables the insertion of a variety of target fragments with no discrimination.

## 5. Discussion

Mutagenesis has been widely used in optimizing and specializing the function of a specific protein in order to obtain a protein for a particular purpose or a designed phenotype of an organism. Saturation mutagenesis is a powerful strategy targeting a selected amino acid or targeting nearly all amino acids of a protein through sequential steps. Application of degenerate oligonucleotides is the straightforward method of saturation mutagenesis. In the present study, partially degenerate oligonucleotides are employed for a completely new purpose in mutagenesis-evaluation of the mutation tolerance of a reporter gene. ZeoR has been identified to be highly tolerable to mutations at the sites tested. As ZeoR had no bias in nucleotide use at each degenerate site, it may be a good candidate reporter gene for the development of assays used in the analysis of enzymatic activity and off-target effects of genetically engineered nucleases.

ZeoR has the ability to kill both prokaryotic and eukaryotic cells. This feature renders it to be a precious reporter gene in genetic engineering including gene subcloning. In addition, target sequences for gene editing enzymes, such as ZFNs, TALENs, and CRISPR/cas9, are highly heterogeneous and the length of targets ranges from 20 to more than 60 nucleotides. Thus, an ideal reporter gene needs to tolerate insertion mutagenesis of relatively long inserts and to not exhibit sequence discrimination.

Oligonucleotides flanking three completely degenerate nucleotides NNN are efficient and simple in saturation mutagenesis of a selected amino acid. However, a long string of N nucleotides is very inefficient in obtaining mutants, mainly because of premature termination due to the high frequency of nonsense mutations (Table 3). Therefore, we employed tandems NNC and NNT to reduce the risk of stop codons in the inserted mutants. The present study has demonstrated that the inserts containing (NNC)_8_ and (NNT)_8_ are efficient in yielding mutants. Sequence analysis further identified no bias in the nucleotides used at the degenerate sites, which was the major argument to be tested by the design. Interestingly, the insertion mutants display variable length of inserts, ranging from adding 4 to 12 amino acids corresponding to the 8 partially degenerate triples in the designed oligonucleotides. The mutants with truncated or expanded lengths from these partially degenerate oligonucleotides demonstrate a new useful feature of the tandem NNC and NNT nucleotides in mutagenesis. These two pieces of evidence, where there is no bias in nucleotides used and no fixed length of the inserts, indicate that ZeoR may be a good reporter gene as expected (Table 1). Further insertion mutageneses including some real targets of TALENs and CRISPR/cas9 confirmed the usefulness of ZeoR (Table 4). As shown in Table 4, all designed mutants were obtained and the drug resistance is maintained when there are no frameshift mutations. This selectivity is important because gene editing can result in a frameshift mutation from the repairing of a double-strand break.

Actually, the ZeoR gene can be broadly employed in the analysis of both enzymatic activities and the off-target effects of gene editing enzymes including ZFNs, TALENs, and CRISPR/cas9. The enzymatic activities can be evaluated either in prokaryotic or eukaryotic cells as zeocin is able to kill both types of cells. When the target gene is subcloned into the ZeoR reporter, cotransform or cotransfection of the reporter gene with the gene editing enzyme-encoding vectors will be a simple and efficient assay for the enzymatic activity evaluation. Similar to the enzymatic activity analysis, off-target can be sensitively studied with the same procedure except for the subcloning of mismatched target or selected “off-target.”

Both tandem NNC and tandem NNT oligonucleotides can avoid the formation of nonsense mutations in the insertion mutants. As aforementioned, these two partial degenerate oligonucleotides are sensitive in testing whether there is a bias in nucleotide use at the degenerate sites. However, significantly more mutants with eight amino acids are added in the products using (NNC)_8_ in comparison to those of (NNT)_8_. Whether this difference is the result of stronger base paring between the NNC and GNN is to be elucidated; however, this observation may indicate that tandem NNT oligonucleotides are more effective for testing the mutability of a target.

In conclusion, the present study tested a new strategy for testing mutability of a target by using partially degenerated oligonucleotides. Both tandems NNC and NNT can be used to screen bias in base selection at the degenerate sites and length discrimination to the inserts. The data may further indicate a higher potential of tandem NNT in mutability studies as compared to tandem NNC. Finally, ZeoR has been screened as a good candidate reporter gene in the development of assays in evaluating the enzymatic activity and off-target effects of gene editing enzymes.

## Figures and Tables

**Figure 1:** Plasmid maps of pZAmpA and pZAmpB. (a) The inserted BaeI site and its nucleotide sequences are marked and illustrated. (b) The detailed subcloning sites and their specific sequences before and after cloning are marked.

**Figure 2:** Chromographic illustration showing the correct sequences of the pZAmpA and pZAmpB plasmids.

**Figure 3:** Chromographic illustration showing the correct sequences of inserts.

**Table 1:** Nucleotides used at the degenerate sites corresponding to the tandem NNT and NNC oligonucleotides in the mutants sequenced.

NNT	Sequence	NNC	Sequence
1	CTTGATGGT	1	GACAACAACGAC
2	CATTTTACTAGT	2	ACCAACAACATCCAC
3	AATTATAATGCTAATGGTCTT	3	CTCAGCTTCCTCCCCTGC
4	AGTACTGATTATGTTAATCAT	4	AACATCTTCAGCGGCGACCGC
5	TCTGATTCTCCTTCTCTTCAT		
6	ACTACTCCTTGTTCTGTTCTT	5	AGCTCCGACGACGGCTTCCCCTTC
7	TCTGTTACTGATCTTCCTATT	6	ATCAACATCCACTGCTTCGGCCAC
8	AGTGATCGTGCTTTTGTTAGT	7	AGCTCCGACGACGGCTTCCCCTTC
9	CCTGCTCGTCGTCGTCATCGT	8	CACACCCTCCGCCCCGGCACCTCC
10	GCTTATTCTCTTGTTGTTCGTCGT	9	CACTGCAGCCTCTCCAACTACTGC
11	GGTGATGTTCGTAGTAATCATGGT	10	AACCACGACACCAACCGCAACTTC
12	GTTGGTTCTCGTCGTATTTGTGTT	11	AGCTCCCCCCCCAACTTCACCGAC
13	TCTCATGTTCCTGCTACTTGTCGTCTT	12	AACCTCCACGACCTCGGCCACTAC
14	ATTGGTGGTGCTCTTCCTACTCATTGT	13	AACCACCACTCCACCTTCTGCCAC
15	CTTCATCGTCCTCCTCTTCCTGTTATT		
16	ATTATTTTTACTGCTTGTCCTTGTATT		
17	TCTCCTCTTAATGTTGGTGGTCGTCCTCGTGTTCGT	14	ATCCACCCCTCCCACTGCGTCGCCCTCTCC

**Table 2:** Amino acids deduced from nucleotides used at the degenerate sites corresponding to the tandem NNT and NNC oligonucleotides in the mutants sequenced.

NNT	Sequence	NNC	Sequence
1	LDG	1	DNND
2	HFTS	2	TNNIH
3	NYNANGL	3	LSFLPC
4	STDYVNH	4	NIFSGDR
5	SDSPSLH		
6	TTPCSVL	5	SSDDGFPF
7	SVTDLPI	6	INIHCFGH
8	SDRAFVS	7	SSDDGFPF
9	PARRRHR	8	HTLRPGTS
10	AYSLVVRR	9	HCSLSNYC
11	GDVRSNHG	10	NHDTNRNF
12	VGSRRICV	11	SSPPNFTD
13	SHVPATCRL	12	NLHDLGHY
14	IGGALPTHC	13	NHHSTFCH
15	LHRPPLPVI		
16	IIFTACPCI		
17	SPLNVGGRPRVR	14	IHPSHCVALS

**Table 3:** Advantage and disadvantage of completely and partially degenerated oligonucleotides in mutagenesis.

Oligo type	Advantage	Disadvantage
NNN	Efficient for saturation mutagenesis	5% chance of creating nonsense mutations

NNT	Tandem triplet can be used to test mutability of a target gene; both the bias of nucleotide use and the length of inserts can be tested	One triplet can be used for saturation mutagenesis when combined with NNG

NNC	Tandem triplet can be used to test mutability of a target gene, but the power may be lower than that of NNT; both the bias of nucleotide use and the length of inserts can be tested	One triplet can be used for saturation mutagenesis when combined with NNG

**Table 4:** Designed mutants keep the zeocin resistance gene in frame.

Size (nt)	Targeted gene	Sequence	A : T : C : G ratio
32	n.a	CTAGAGATATCGTCGACCTGCAGAAGCTTCCG	8 : 7 : 9 : 8
33	n.a	CCTAGAGATATCGTCGACCTGCAGAAGCTTCCG	8 : 7 : 10 : 8
111	n.a	CCTAGAGATATCGCATGCCTGCAGGTCGACTCTAGAGGATCCCCGGGTACCGAGCTCGAATTCACTGGCCGTCGTTTTACAACGTCGTGTCTGGGAAAACCCAAGCTTCCG	24 : 25 : 33 : 29
112	n.a	CCTAGAGATATCGCATGCCTGCAGGTCGACTCTAGAGGATCCCCGGGTACCGAGCTCGAATTCACTGGCCGTCGTTTTACAACGTCGTGTCTGGGAAAACCCCAAGCTTCCG	24 : 25 : 34 : 29
51	CCR5-1-3N	TGCATCAACCCCATCATCTATAGATCTGTCGGGGAGAAGTTCAGAAACTAT	16 : 13 : 12 : 10
52	CCR5-1-3N+1	TGCATCAACCCCATCATCTATAGATCTGTCGGGGAGAAGTTCAGAAACTATC	16 : 13 : 13 : 10
39	EGFR 15-1-3N	AAGCTGGCTTTCGGAGATGTTTTGATAGCGACGGAATTC	9 : 12 : 6 : 12
40	EGFR 15-1-3N+1	AAGCTGGCTTTCGGAGATGTTTTGATAGCGACGGCAATTC	9 : 12 : 7 : 12
42	EGFR 18-1-3N	AAGCTGTCGCTATCAAGGAATCGAAAGCCAACAAGGCAATTC	16 : 7 : 10 : 9
43	EGFR 18-1-3N+1	AAGCTGTCGCTATCAAGGAATCGAAAGCCAACAAGGCAAATTC	17 : 7 : 10 : 9
